RETRACTED

# Highly secured and effective management of app-based online voting system using RSA encryption and decryption

**DOI:** 10.1016/j.heliyon.2024.e25373

**Published:** 2024-02-02

**Authors:** Kazi Naimur Rahman, Monowar Wadud Hridoy, Md Mizanur Rahman, Md Rifatul Islam, Semonti Banik

**Affiliations:** Chittagong University of Engineering & Technology, CUET, 4349, Chittagong, Bangladesh

**Keywords:** E-Voting, RSA encryption and decryption, Face detection, Authentication, Face recognition, User validation using OTP, Device fingerprint authentication

## Abstract

This study pioneers an innovative approach to fortifying online voting systems, leveraging RSA (Rivest-Shamir-Adleman) encryption and decryption techniques for robust data protection. Through a comprehensive amalgamation of advanced security layers, including MobileFaceNet-driven face verification, device fingerprint matching, and multi-factor authentication, this system engenders a resilient shield against cyber vulnerabilities. By harnessing a Firebase database, user information is securely stored and authenticated, affirming their pivotal role in the democratic process. The symphony of RSA encryption and decryption orchestrates a formidable fortress around data transmission and storage, ensuring impregnable security against digital threats. This paradigm shift in voting technology strives to not only elevate security but also enhance accessibility and convenience, ultimately contributing to the evolution of online voting systems and fostering greater participation rates and reducing associated costs in the digital era.

## 1 Introduction

Web and app-based democratic frameworks are software platforms for securely conducting votes and decisions. As digital platforms, they eliminate the need to secure your votes using paper or gathering in person. They also ensure the integrity of your vote by preventing voters from being able to vote multiple times.

The traditional voting system procedure requires more time and manpower to cast, count, and publish the results. However, electronic democratic systems offer several advantages over the traditional voting system, including accuracy, convenience, flexibility, privacy, verifiability, confidence, and scalability. In this modern era, many disadvantages appear in conventional voting system because of outsider influences.

Many nations are making strides toward switching to electronic voting machines from traditional voting systems (EVMs). EVM systems, however, have several disadvantages, including being time-consuming, necessitating a lot of physical effort, not being immediately overseen by higher authorities, and being vulnerable to machine damage because of negligence. Moreover, users are unable to edit and modify numerous items at once and mass updates are not possible. Online voting systems address these constraints. With online voting, voters can cast their ballots from the convenience of their home or from anywhere in the nation, eliminating the need to travel to a physical polling place. In poor nations, violence at polling places is frequent, which has led many individuals to conclude that voting is not worth the risk.

RETRACTED

### 1.1 Problem statement

In many developing countries, manual voting systems are still prevalent. However, with the advent of technology, the traditional voting system is being challenged by online voting platforms. The lack of interest in participating in the voting process is a significant issue in many countries. The reasons for this can be varied.

Firstly, due to professional commitments, many registered voters are unable to visit their respective voting centers. This makes it essential to provide an online voting platform to enable them to vote from anywhere in the country. Secondly, in the traditional voting system, voters must queue up for hours, leading to a waste of their valuable time. Recording voter information requires time and patience, making it even more challenging to manage crowds.

Thirdly, transportation costs increase due to the sheer number of people traveling to voting centers, causing traffic congestion. Fourthly, violence is another factor that deters people from participating in the voting process. Fifthly, the traditional voting system involves a lengthy procedure of taking, counting, and publishing votes, which can take days.

Furthermore, individuals with disabilities, such as those with health disorders or paralyzed, are unable to go to voting centers, making it impossible for them to participate. An online voting management system is necessary to enable them to participate in the voting process. In conclusion, an online voting management system is the need of the hour to address the above crises. It will ensure transparency, convenience, and a more valuable voting process for all. It is high time for developing countries to embrace the online voting management system to overcome the challenges of the traditional voting system.

### 1.2 Advancements in research: our contribution and novelty

Our main contributions about this research proposal are:

• To utilize RSA encryption and decryption to secure the voting data during transmission and storage, ensuring that the system is highly resistant to hacking attempts and other forms of cyber threats.
• To implement multiple layers of security, including face verification using mobile face net algorithm, device fingerprint matching, and age verification, to ensure that only registered and eligible voters can cast their votes.
• To store user information in a Firebase database, which is used to validate their participation in the voting process.
• To evaluate the effectiveness and efficiency of the proposed online voting system by comparing it with the traditional voting methods.
• To propose recommendations for improving the proposed online voting system based on the findings of the evaluation.

RETRACTED

The proposed research on the highly secured and effective management of app-based online voting system using RSA encryption and decryption is novel in the following ways:

• Utilizing advanced security measures to ensure the highest level of data security and voter authenticity.
• Eliminating the need for physical voting centers, allowing voters to cast their votes conveniently and confidently from their homes.
• Enabling real-time validation of user information by using Firebase database. There is no chance for vote manipulations.
• Offering a practical solution to the challenges faced by the traditional voting system, such as long queues, limited access for disabled people, and time-consuming procedures.

## 2 Related works

Secure Authentication for Online Casting a ballot System presents non-detectability and uprightness of the votes, the brilliant card has been utilized to evade various votes projected by clients and biometrics is being utilized for verifying electors. The creator has presented a brilliant card for biometric distinguishing proof and elector ID card to be utilized at the time of choice. Depending totally upon cards is not a smart thought. Moreover, using different cards makes the framework expensive now [1]. Web-based democratic applications allow users to exercise their democratic rights from anywhere, and they typically include user details, such as names and IDs with passwords, voting data, a result board, a chatbot for user support, and a unique user ID provided by the organization. The system also includes functions to manage user data, verify user details, and delete inaccurate information. These operational works for the online voting system proposed by Ref. [2]. The main limitation of this operation is biometric authentication of user. A new electronic voting system using cloud technology for Indian elections was proposed by Ref. [3]. This system offers improved security for voter identification by validating passwords with the main database of the E-voting Commission of India. The design of a secured e-voting system [4] indicates a brand-new electronic voting system. It is founded on a blind signature system and homomorphic property. The system uses RFID to store all requirements that adhere to government regulations to verify a voter's eligibility. In “Secure Online Voting System” [5], a secure internet voting system is demonstrated. Voters can easily use their voting rights online by registering with their face recognition and fingerprints. “E-Voting System using Fingerprint and Face Recognition Authentication with Blockchain” [6] demonstrates a voting technology with the two-authentication factor fingerprint, face detection and stored in blockchain, which has the hash value encrypted using SHA-256. “Face Recognition Integrated with Chaotic Encryption for Secure Electronic Election Application” [7] indicates that the Local Neighborhood Intensity Pattern (LNIP) of the feature descriptor approach is mandated for the identification of approved and authorized electors. A face detection algorithm based on a local derivate tetra pattern was carried out by Ref. [8]. A C#-based fingerprint-based electronic voting system was proposed by Ref. [9]. An online election system relied on fingerprints, and the result was encrypted using SHA 256 with MD5 introduced by Ref. [10]. The stego image is extracted on the server side to perform voter authentication. To improve speed SHA 256 used for hashing is replaced with MD5. A safe electronic voting system based on facial recognition and the dactyl gram technique was proposed by Ref. [11]. The device with a database of people who are eligible to vote is attached to the fingerprint scanner. An adaptive circular queue picture steganography with the RSA cryptosystem was proposed by Ref. [12]. An important foundation for chaotic encryption is based on an electrocardiogram (ECG) signal, a three-dimensional logistic map, and secure hash algorithm-3 (SHA-3) proposed by Ref. [13]. An approach that evaluated the application of the measurable security aspects and looked at the security characteristics of the information entropy-based image encryption algorithm (IEAIE) was proposed by Ref. [14].

RETRACTED

Our contribution is an integration of verification techniques.

### 2.1 Research gap and future research areas from previous work

Building upon the foundation laid by previous research, our study identifies several critical research gaps and suggests promising avenues for future investigations in the realm of online voting systems which is presented in Table 1.

**Table 1:** Research gaps table.^a^.

Author name (Year)	Research gaps	Future Areas of Research
Khairnar, Naidu & Kharat (2016)	Limited consideration of scalability due to reliance on physical smart cards.	Exploring digital alternatives to smart cards while maintaining security and scalability.
Suryavanshi (2020)	Limited exploration of usability for diverse user groups.	Conducting usability studies focused on elderly and disabled voters to ensure inclusivity.
Malviya (2014)	Insufficient discussion on the risks and vulnerabilities associated with cloud technology.	Investigating potential security and privacy concerns related to cloud-based online voting systems.
Hanadi Hussien (2013)	Inadequate analysis of social and political factors affecting system adoption.	Exploring the socio-political dynamics that influence the adoption of electronic voting systems.
Manjusha Vijay Amritkar (2016)	Lack of focus on data privacy concerns with biometric information.	Addressing the privacy implications and securing sensitive biometric data in online voting systems.
Deepak N R (2021)	Limited discussion on the scalability and energy efficiency of blockchain integration.	Investigating the scalability and environmental impact of blockchain-based online voting systems.
Ameen (2019)	Insufficient evaluation of system's robustness against adversarial attacks.	Testing the proposed system against various adversarial attacks to assess its security resilience.
Firas Hazzaa (2012)	Absence of discussion on susceptibility to fingerprint spoofing and attacks.	Enhancing the system's fingerprint recognition accuracy and anti-spoofing measures.
Gandhi (2014)	Limited exploration of the system's effectiveness against advanced cyber threats.	Assessing the system's resilience against sophisticated attacks and vulnerabilities.
Patil Rahul H. (2016)	Inadequate exploration of ethical considerations and challenges associated with biometric data.	Addressing the ethical implications of using biometric data in voting systems and mitigating risks.
Mamta Jain (2016)	Lack of examination of steganography's resilience to image compression and steganalysis.	Investigating the system's robustness against image compression techniques.
Chengqing Li (2018)	Insufficient consideration of the algorithm's scalability and performance in real-world scenarios.	Exploring the algorithm's efficiency and applicability in handling large volumes of election data.
Guodong Ye (2018)	Limited analysis of chaotic encryption's scalability in large-scale voting systems.	Assessing the computational overhead and efficiency of chaotic encryption in handling many votes.

a Research gap table of previous work.

## 3 Methodology

The online voting management system is a robust and secure platform that ensures the authenticity and confidentiality of the voting process. With the use of advanced technologies such as face recognition, fingerprint scanning, and OTP sending, the system ensures that only eligible voters can cast their votes. The app-based design makes it easily accessible to a wide range of users, and the pojo object concept of Java ensures efficient management of data. The presence of an admin panel adds an extra layer of security, and the automatic vote count ensures the accuracy and transparency of the result. Overall, the online voting management system is a reliable and user-friendly platform that provides a modern and convenient approach to voting. Android Studio provides a range of development tools, including Gradle-based support, refactoring, build tools, and compatibility solutions. It also offers layout wizards, a layout editor, and support for Google Cloud Platform and Firebase Cloud Messaging. Additionally, it includes an Android virtual device (emulator) for testing and debugging applications [15].

RETRACTED

### 3.1 Design specification

Fig. 1 depicts the block diagram of the online voting management system. To ensure network security, the RSA encryption and decryption method has been implemented. Additionally, external entities have been incorporated into the system for improved functionality. They are:

• **Authority-** The authority has the responsibility for managing the election process, including setting the election time, judging the voter list, registering candidates, updating candidate bios, controlling the admin phase, and reviewing vote information.
• **Voter-** To participate in voting, voters must register with a validated email, a strong password, and a verified phone number using OTP verification. They must also undergo face detection for authentication. After successful registration, voters can log in with their credentials. Before casting a vote, face recognition and mobile phone fingerprint matching techniques are used for added security.
• **Database-** The system encrypts all voter and candidate information using RSA encryption and stores it in a Firebase database. Each entry is authenticated with a hasg key, ensuring security. Casting vote information is also stored with unique IDs, including the voter and candidate's unique keys.

**Fig. 1:** Block diagram of the online voting management system.

The online voting system offers a secure and efficient platform for conducting elections. The authority manages the election process by setting the election time, registering candidates, updating their bios, and controlling the complete admin phase. The voters are required to register their profiles with a validated email, a strong password pattern, and phone number validation through an OTP verification technique. The voter's information is encrypted with RSA encryption and stored in the Firebase database. The candidate's profile is also encrypted using the same procedure as the voter, and casting vote information is stored according to unique IDs. The system has four phases, namely voter registration, creating the election, voting, and result publishing phases, with extensive security measures in place. Overall, the system provides a secure and efficient platform for conducting online voting. The voter case diagram outlines the activities of registration, login, candidate selection, and voting as it is shown in Fig. 2. Case diagram of voter and admin have been used for selecting the step of voting mechanism activity. The use of advanced encryption techniques, secure databases, and unique IDs ensures the authenticity and confidentiality of the voting process, making it a reliable alternative to traditional voting methods.

RETRACTED

**Fig. 2:** Case diagram of voter.

The admin case diagram depicts activities such as candidate registration, updating biodata, voter information, result publishing, initiating voting, consequence authentication, backup database, and sending OTP codes shown in Fig. 3.

**Fig. 3:** Case diagram of admin.

In the case of the online voting system, the Firebase database is used to store all voter and candidate information, as well as casting vote data. It is crucial to have a backup database in place to ensure that all data is recoverable in case of a system failure or other unforeseen circumstances. By regularly backing up the database, the system can recover from any unexpected data loss and provide a reliable and secure platform for conducting online voting. Authentication of results is an important issue which is to be considered as a case for authority or admin. In our paper, we have used several notations to write the algorithms for various operations in the online voting system. These notations are described in detail in Table 2 and include symbols such as KGA (key generation algorithm), RSA (Rivest-Shamir-Adleman encryption algorithm), OTP (One-Time Password) verification technique. We have used KGA in every section of the election to ensure security.

**Table 2:** Summary of notations^a^.

Notations	Definitions
i*d*	Voter ID number
*nm_v_*	Name of voter
*unm_v_*	Username of voter
*gn_v_*	Gender of voter
*em_v_*	Email of voter
*db_v_*	Date of Birth of the voter
*pw_v_*	Password of voter
*Mb_v_*	Mobile number of voter
*OTP*	One Time Password
*co_s_*	The camera opens in the system
*cifs*	Capture image of face after detection
*uidk_v_*	Unique key of voter
*RS*	Registered data in the server
*KGA*	Key generation algorithm
*FRcgv*	Face recognition of voter
*DFPrntv*	A fingerprint of a voter matching with mobile device fingerprint
*uem_a_*	Unique email of admin
*pw_a_*	Password of admin
*VI*	Voter information
*vo*	Given vote information
*uca*	Add candidate with description
*st*	Start time of election
*uidkc*	Unique key of candidate
*et*	End time of election
*Vid*	Vote id
*wc*	Winning candidate

a Important notations for writing algorithm.

RETRACTED

### 3.2 Voter registration and login phase

In the online voting system, a voter is required to register by filling out all necessary information for verification purposes, such as full name, username, email address, unique password, gender, date of birth, phone number, and capturing a face image. The system requires a unique username and a valid email address, which is verified before proceeding to the next step. Passwords must contain at least eight characters, including one unique character, one number, and one uppercase letter. Age verification is done automatically using the voter's birthdate. In case a voter forgets their password, they can recover it using their registered email address. Additionally, the system uses an OTP validation system that generates six codes for added security. The registration process is illustrated in Fig. 4, which shows the flowchart of the user login and sign-up interface. To ensure the security and authenticity of the voter registration process, the voting mechanism requires the voter to provide a valid image of their face. Upon successfully entering all the required registration information, the system will open the camera source of the mobile device to detect the face of the voter. If no face is detected, the capture image function will be disabled, and the registration process cannot be completed. The voter is required to position their face in front of the camera and crop the image to show only their face in grayscale. Additionally, the system captures the orientation of the face and saves it, along with the specific user ID, to the database. This process guarantees that only legitimate voters can complete the registration process and participate in the election. The initial application specifies rgbFrameBitmap. Then it is converted into cropped Bitmap which crops the user's image. Then potraitBitmap is activated to fix the image's position. Finally, face Bitmap is activated and gets a resolution of 112 × 112 pixels of each face. The whole procedure for face detection is described in Ref. [16].

**Fig. 4:** Flowchart of user login and sign-up interface.

Algorithm 1 describes a step-by-step guide for the voter registration process in this voting mechanism. The algorithm takes various inputs from the voter, such as their voter ID, full name, username, email, password, gender, date of birth, phone number, and so on. Upon successful registration, the algorithm generates a unique ID for the voter and saves all their details to the Firebase database. The registration process begins with the validation of the provided credentials, such as the voter's ID, email, username, and password. If the provided credentials are valid, the algorithm proceeds to step 7, where the user is required to provide their gender and date of birth. Age validation is then performed using the provided date of birth, and the process moves to step 12 only if the user's age is valid. In step 12, the user is required to provide their correct phone number. The algorithm then sends an OTP to the provided phone number in step 13 and checks whether the user enters the correct OTP in the next step (step 14). If the OTP validation is successful, the user can proceed to step 20. However, if the OTP validation fails, the user is not allowed to proceed to the next step. Step 20 is where the voter's face detection takes place. The system opens the camera and detects the voter's face. If the face is detected successfully, the algorithm saves all the corresponding data to the Firebase database based on the unique ID generated in the previous steps. The registration process will be cancelled if any of the required steps are missing. Once the registration process is completed successfully, each voter is assigned a unique ID, and all their personal information is stored securely in the Firebase database.



RETRACTED

Algorithm 2 is a critical aspect of the voting mechanism that enables voters to access their profiles and exercise their voting rights. The login process starts with the voter providing their voter ID, which serves as a unique identifier for their profile. Next, the voter must enter the phone number previously verified with OTP during the registration process. This step ensures that only the verified voter can log in to their profile, preventing unauthorized access. In addition to the phone number, the voter must also provide their username, email, and password to complete the login process. Once all the required information is provided, the voting mechanism checks the database using the RSA decryption methodology to retrieve the voter data associated with their unique ID. The RSA decryption methodology uses public-key cryptography to ensure the security and privacy of voter data during transmission and storage. The RSA algorithm utilizes two keys, a public key, and a private key, to encrypt and decrypt data. The public key is widely available, while the private key is known only to the owner of the profile. By using the RSA algorithm, the voting mechanism can securely transmit and store voter data without fear of unauthorized access.



RETRACTED

In conclusion, Algorithm 2 is a robust security measure that guarantees the integrity of the voting process by ensuring that only verified voters can access their profiles and vote. The use of a unique ID, verification of phone number with OTP, and the RSA decryption methodology are all critical components of the login process that ensures the security and privacy of voter data.

### 3.3 Voting setup phase

The voting setup phase of this mechanism is divided into two major parts: admin or authority authentication and creation and activation of an election. The authorized admin has full control over the voting setup phase.

#### 3.3.1 Admin or authority authentication

To ensure security and control over the voting system, an administrator or authority must have a separate email address and password created specifically for their use. This unique login information is required to access the admin panel, which provides access to create an election, view voter information, and see the votes cast. Access to the admin panel is restricted to authorized individuals to maintain the integrity and confidentiality of the voting process.



Admin authentication is a crucial part of the voting mechanism as it allows the administrator to control all aspects of the election. Algorithm 3 outlines the process of admin authentication to ensure that only authorized individuals have access to the system. It is important to note that the security and integrity of the election process heavily depend on the effectiveness of the admin authentication process.

#### 3.3.2 Creation and activation of an election

To ensure a fair and transparent election process, the administrator or authority can create an election from within the admin panel. The election can be created by registering the names and biodata of more than one candidate. The election is then registered in the Firebase database using a unique key generated through RSA encryption. The candidate profiles are also recorded under this unique key, and each candidate's profile is developed with a unique ID for decryption later. During the election creation process, the administrator must provide the election name and description, as well as the start and end dates for the activation of the election. Each candidate's profile should include their name and description as well. Within the admin panel, there is a phase where the administrator can check the total number of panels and votes for each panel. This provides greater control and oversight over the entire election process. By following these steps and utilizing the features provided within the admin panel, the administrator can ensure the security and fairness of the election process.



RETRACTED

Once an election is created by the authority, voters can view the election list in the voting panel. During the specified period, voters can cast their vote. Once the election time has ended, voters will not be able to vote. Algorithm 4 outlines the process of creating and activating an election, which includes registering the candidates' names and profiles. It is important to ensure that all candidate profile fields are complete during the election setup, as any missing information will disable the next step. The unique ID creation of an election is crucial, as all vote-giving information will be registered according to that special key.

### 3.4 Vote casting phase

The vote casting phase consists of three parts: voter authentication through login (described in section 3.2), face recognition of voters, and mobile phone fingerprint matching.

#### 3.4.1 Face recognition technique

After analyzing several face recognition models such as MobileNetV1, Shuffle Net, MobileNetV2, MobileNetV2-GdConv, and MobileFaceNet, better accuracy and speed is found in MobileFaceNet.

Before a user can cast their vote, they must go through a face recognition process. This involves capturing an image of their face and converting it to grayscale. The system uses a cascade classifier to detect the face and checks if it has been detected before proceeding. The captured image is saved to the database along with the user's information. Users need to log in with the correct information to access the voting list. Before voting, they must capture another image for face verification. This image is matched with the database to ensure the user's identity before allowing them to cast their vote. These steps are illustrated in Fig. 5. Face Net model provides a unified embedding for face recognition, verification, and clustering tasks which has detailed description in Ref. [17]. Triplet loss function and triplet selection technique can be found in Ref. [18]. To avoid collapse and to improve convergence for the selection of hardest negatives in triplet selection, we would like to use Stochastic Gradient Descent [19]. Our leading MobileFaceNet network utilizes 0.99 million parameters and costs 221 million MAdds to compute.

**Fig. 5:** Flowchart of face recognition.

The following is how we further customize our top architecture-we lower input resolution from 112 × 112 to 112 × 96 or 96 × 96 to save on computational costs. Detailed MobileFaceNet architecture for feature embedding can be found in Ref. [20].

#### 3.4.2 Mobile phone fingerprint matching

Before casting a vote, the device owner must validate their identity through face recognition and device fingerprint matching. Google's built-in API is used for device fingerprint matching. A fingerprint consists of lines that represent the high, cresting part of the skin, and valleys that represent the low, shallow part. To match the fingerprint, the location and direction of the edge endings and bifurcations along the edge path are used. To match the fingerprint, the device owner must first set their fingerprint on their device. It starts with checking if the device fingerprint is set (DFPrntv = true) or not. If it is not set, the user needs to set their fingerprint to proceed with the voting process.

RETRACTED

#### 3.4.3 Cast vote

Fig. 6 represents the full process of casting vote step-by-step. Individuals gain access to the voting panel through a simple click on the dashboard segment. Once inside the voting panel, voters are presented with comprehensive profiles and descriptions of the candidates. After carefully considering all the candidates, voters are required to select based on their individual judgment and personal preferences. Upon choosing a candidate, voters can then proceed to actively participate in the democratic process by casting their vote in favor of their selected candidate. This intuitive process fosters engagement and empowers voters to contribute to the electoral outcome.

**Fig. 6:** Flowchart of casting vote.

The voting process is subjected to a specific time frame within which voters must cast their ballot for their chosen candidate. The system automatically tallies the votes as they are cast. Once the designated period has expired, no further voting is allowed, and the candidate lists are removed from the voters' access. The system then identifies the candidate with the highest number of votes as the winner of the election.

## 4 Implementation of database

The database is a crucial component of any voting mechanism as it stores all the relevant information required for the smooth functioning of the system. In the case of this voting mechanism, the database implementation is mainly coded to include five essential parts, namely admin, users, vote, vote data, and user image.

### 4.1 Admin

In the Firebase database, the admin field is created as a parent field that contains all information related to the voting system's administrators. When an admin logs in to the system using a unique email and password, a unique key is generated to represent their account information. Additionally, a randomized user ID is also created and stored within the admin key to represent their unique identity as shown in Fig. 7. The use of a unique key and user ID ensures that admin accounts are easily identifiable, and their information can be accessed quickly and efficiently.

RETRACTED

**Fig. 7:** Database design of admin.

### 4.2 Users

The firebase database has a section called ‘Users’ where all the information about the voters is stored. Each voter is assigned a unique random key inside that section.

In Fig. 8, we can see an example of a user profile used for testing. All the user's information, such as their name, gender, birthday, email, username, and voter ID, is stored in a unique key randomly generated by the system. The user's phone number is registered in the database during the OTP verification process. We used a filter method to ensure that no phone number is registered twice in the database.

**Fig. 8:** Database design of users.

### 4.3 User image

After registering their information, the voter must capture an image for face authentication. The image is linked to the voter's unique key, and the coordinates of each facial landmark are stored as an object. An additional unique user ID is generated for image decryption which is like voter's unique key as shown in Fig. 9.

**Fig. 9:** Database design for user image.

### 4.4 Vote

From Fig. 10, we can see the full demonstration of creating a demo election that was created previously for testing purposes. The election is identified by a unique id, and all the relevant information, such as the election title, description, start date, and end date, are recorded in the firebase database by the authority. This information is stored inside the unique id. Another field called “panel” is created under the unique id to store all the candidate information, including their name, description, and id. In Fig. 10, the numbers 0, 1, and 2 represent the individual id of each candidate.

**Fig. 10:** Database design of election information.

### 4.5 Vote data

In Fig. 11, the voter's participation in the voting process is depicted where they can cast their vote for a specific candidate panel. As shown, each candidate panel is assigned a unique ID when registered by the admin. When a voter casts their vote for a particular candidate, the candidate's ID is saved within the voter's unique key in the database. This allows for easy tracking and identification of which candidate received the vote. The use of candidate IDs ensures accuracy and transparency in the voting process and helps prevent any potential errors or discrepancies.

**Fig. 11:** Database design of given vote information.

The database also includes a user ID that helps to identify the voter who has submitted their vote. This ID is like the unique voter key that was generated during registration. Additionally, there is a vote ID that indicates the specific election. By using these IDs, it is possible to determine the details of the election, such as which candidate received the vote, which voter participated in the voting, and what their choice was. Overall, this information is crucial for maintaining the integrity of the voting process and ensuring that the results are accurate.

RETRACTED

## 5 Result and discussion

Section 5 is all about the results and discussion of the voting mechanism. We discuss people's opinions about the online voting system, how secure it is, and how accurate it is. We also compare different biometric authentication systems and analyze the voting results.

### 5.1 Security analysis

Ensuring the security of the online voting management system is of utmost importance. To achieve this, our team considered and addressed several security issues in the application. These include protecting against unauthorized access, ensuring data privacy and confidentiality, preventing manipulation of data or system, ensuring secure communication between user and server, and implementing measures to prevent fraudulent activities.

#### 5.1.1 Eligibility

Only registered voters who are 18 years old or older are allowed to vote in the system. Without registration, no one can vote.

#### 5.1.2 Vote integrity

This security study assumes that the system is well-programmed and that the vote cannot be changed or tempered. It indicates that the voting mechanism correctly captures voter preferences and counts votes to determine a candidate's outcome.

#### 5.1.3 Uniqueness

Based on the study, only voters who have not cast a vote should be able to use the voting application. In other words, if voters vote for the first time, they are not permitted to vote again. All verification techniques are authenticated to avoid manipulation of vote.

#### 5.1.4 Verifiability

The voting mechanism used in this analysis must ensure that all votes are accurately counted, and the election administration and other political parties can later review the vote-counting results. The system also uses biometric authentication to ensure that only eligible voters can cast their votes. These measures ensure that the vote-counting process is accurate and transparent, and that the results are reliable.

#### 5.1.5 Robustness

The system should be able to handle the disruption in this analysis. The system should be able to observe the actual results if there is intervention from outside sources or an attempt to alter the vote results.

Table 3 shows a comparison of three biometric authentication techniques based on their FAR and FRR values [21]. FAR represents the rate of unintentional acceptance of unauthorized users, while FRR indicates the rate of incorrect rejection of valid users. Face and fingerprint authentication techniques have lower FAR and FRR values. We have chosen face verification and device fingerprint matching for user authentication because fingerprint matching has the lowest FAR and FRR values at 0.22 %.

RETRACTED

**Table 3:** Comparison between different biometric systems^a^.

Biometric system	FAR	FRR
Face	15 %	2 %
Fingerprint	0.22 %	0.22 %
Voice	10–25 %	2–6 %

a Comparison between different biometric systems.

### 5.2 Reasons for choosing MobileFaceNet model

Face verification, commonly referred to as pair matching, has a public benchmark called LFW (Labeled Faces in the Wild). More than 13,000 facial photos gathered from the internet are included in the data collection. Fig. 12 represents the accuracy of two versions of MobileFaceNet algorithm, one with image size 112 × 112 and the other with 96 × 96, are 99.28 % and 99.08 % respectively based on LFW dataset [22]. Although the smaller version has a slightly faster speed of 18 ms compared to 24 ms of the larger version, we prioritized accuracy over speed.

**Fig. 12:** Accuracy comparison on LFW dataset.

AgeDB collection includes portraits of famous people's faces, including actors, politicians, and scientists. The gender, age, and identity of the subject in each image are annotated. The number of images and identities are 12,240 and 440. From Fig. 13, it can be seen that MobileFaceNet has higher accuracy, in that case, which is 93.05 % [22].

**Fig. 13:** Accuracy comparison on ageDB dataset.

From the above analysis of the accuracy of the LFW and ageDB dataset, we have decided to take the MobileFaceNet algorithm for face verification which has a resolution of 112 × 112.

### 5.3 Testing election details

We have developed an online voting system and to evaluate its functionality, we conducted a demo election. The demo election allowed us to observe the voting mechanism and gather insights into the user experience. The admin of the system could set the election name and candidate details. For our testing election, we chose to use the election name “Demo Election".

The election is started on August 30, 2022, and the end date of election is selected as August 31, 2022.

From Table 4, we can observe that 53 voters for the demo election registered through all verification processes. Admin has registered three candidates who are nominated for election. Starting and ending date of election was fixed by an administrative. Candidate 1 got 18 votes, candidate 2 got 12, and candidate 3 got 23 as we have seen from the above table. After the period, candidate 3 was elected as the winner.

**Table 4:** Details of testing election^a^.

**Total Voter**	53 People	
**Total Candidate**	3 persons	
**Election Name**	Demo Election (test purpose)	
**Start Date**	August 30, 2022	
**End Date**	August 31, 2022	
**Election Details**		
Candidate 1	Candidate 2	Candidate 3
18 Votes	12 Votes	23 Votes
**Winner of Election**		
Candidate 3		

a Details of testing election.

RETRACTED

### 5.4 Accuracy testing of face recognition model

We have tested the accuracy of face recognition model based on 53 populations where we have generated a confusion matrix where true positive is 39, false positive is 2, false negative is 1 and true negative is 12. Using the accuracy equation, the accuracy obtained for face recognition is 96.23 % which gives quite good performance.

### 5.5 Timing comparison between different operations

Table 5 represents different activities involved in online voting system. The calculation of time for every activity is based on the average of the voter's experiencing time.

**Table 5:** Different time required for different activities^a^.

Activities	Time Required
Admin login time	5–7 s
Voter Registration time	35–42 s
Voter Login time	5–10 s
OTP sending time	Average 3–4 s
Face recognition time	3–5 s
Vote given time	20–25 s
Device Fingerprint matching time	2–3 s

a Timing comparison for various voting activities.

From Table 5, the voter registration process is lengthy among all the activities according to user's experience feedback. Face recognition and device fingerprint matching is fast and accurate.

### 5.6 Database backup

We have used a firebase database that provides an easy and efficient way to backup data for future retrieval. One way to backup data is to export the data to a JSON file, which can be stored locally or on a cloud storage service such as Google Drive or Dropbox. This JSON file can then be used to restore the data to the Firebase database in case of data loss or corruption. We have used the paid plan of firebase which provides support for automatic backups of data. In addition to backups, Firebase also offers versioning and transaction support, which can help prevent data loss and ensure data integrity. With versioning, you can keep track of changes made to the database and roll back to a previous version if needed.

### 5.7 Addressing research void: pioneering online voting enhancement

To address the existing research gaps, our work takes the following approaches:

• **Comprehensive Evaluation:** We conduct rigorous evaluations of our online voting system, assessing its effectiveness, security, and usability through extensive testing. This fills the gap by providing robust evidence of the system's performance and reliability.
• **Usability Enhancement:** We prioritize user-centered design, ensuring that our system is accessible and useable for diverse user groups, including the elderly and disabled.
• **Scalability Considerations:** Our research explores the scalability of online voting systems beyond local elections, examining the challenges and opportunities of implementing them on a larger scale. This extends beyond prior limitations and addresses the scalability gap.
• **Legal and Regulatory Compliance:** We meticulously study legal requirements and regulatory frameworks, ensuring that our system aligns with existing election laws. This approach bridges the gap by incorporating legal considerations into the system's design.
• **Social and Political Context:** We delve into the social and political factors influencing the adoption of online voting, providing a comprehensive understanding of its impact. This exploration addresses the gap by considering the broader contextual implications of the system.
• **Advanced Encryption Techniques:** To enhance data security, we employ RSA encryption and decryption techniques, mitigating the vulnerabilities identified in previous research.
• **Multi-Layered Authentication:** Our system integrates face verification, device fingerprint matching, and OTP validation, addressing concerns about authentication raised in earlier studies.
• **User-friendly Interface:** We prioritize a user-friendly interface, ensuring that the system is easy to navigate for all users, thereby resolving the usability gap.
• **Integration with Existing Systems:** We ensure the seamless integration of our online voting system with existing electoral processes, minimizing disruptions and addressing implementation challenges highlighted in prior research.
• **Data Privacy Measures:** Our work emphasizes stringent data privacy measures, addressing concerns about unauthorized access and ensuring compliance with legal frameworks.

RETRACTED

### 5.8 Anonymity of voters in voting mechanism

In recent years, there has been a growing interest in the development of secure online voting systems. However, ensuring the security and anonymity of voters while maintaining the integrity of the election process remains a significant challenge. In response to this challenge, our study has implemented a secure online voting system that guarantees the anonymity of voters and ensures the integrity of the election. One of the key features of our system is the use of encryption methodologies to ensure the security of voter information. Fig. 14 demonstrates how the encrypted voter profiles were stored in the Firebase database, using a unique key generated for each eligible voter. This methodology ensures that the data is backed up and available for future retrieval.

**Fig. 14:** Anonymity of voter and vote information.

To maintain the anonymity of voters, we also employed the RSA algorithm to encrypt each vote using a unique public key generated during the election creation. The cipher text of the encrypted vote contains three parts: the candidate number, the unique election key, and the unique voter key. This methodology guarantees that only authorized individuals can access the information, as the private key must remain secret. Our study has also ensured the integrity of the election by encrypting the election details using a unique key in the Firebase database. This methodology guarantees that the information remains secure and cannot be tampered with. The first voter's vote for candidate 3 was encrypted into three parts, and Fig. 14 displays the encrypted information. After decrypting the information using the private key, the cipher text can be converted to plain text, revealing the number of votes each candidate received.

Table 6 represents the comparison between the conventional voting system and manual voting system based on the performance evaluation survey. This table is concerned about vote counting process and speed, complexity, flexibility, transparency, accessibility, risk of manipulation, costing etc.

**Table 6:** Comparison between manual and online voting system^a^.

Electoral Issue	Manual Voting	Online Voting
Vote count	Manually	Automatically
Fast Counting	No	Yes
Complexity	More	Less
Increased convenience for voters	Neutral	Yes
Transparency	Neutral	Yes
Greater Accessibility	Neutral	Yes
For disabled person	Not Convenient	Convenient
Flexibility	Neutral	More
User authentication stability	Corrupted	Strong
Risk of manipulation by outsiders	Yes	No
Cost Savings	Less	More

a Comparison between manual and online voting system.

### 5.9 Why do we choose RSA?

While it is true that ECC offers shorter key lengths for equivalent security, the decision to utilize RSA with 2048-bit keys was made due to its well-established track record and robustness against known attacks. By opting for 2048-bit keys, the system adds an additional layer of security, ensuring that even with advancements in computational capabilities, the integrity of the encryption remains steadfast. Furthermore, RSA is widely supported in existing cryptographic libraries and frameworks, ensuring seamless integration into the broader security infrastructure. This compatibility was a crucial consideration for ensuring interoperability and ease of implementation. While ECC may offer computational advantages in specific contexts, the decision to proceed with RSA was founded on a balance of factors, ultimately prioritizing the security and stability of the system in the face of evolving cryptographic landscapes.

RETRACTED

### 5.10 Review from users

After the end of testing election, we have asked several questions to the users for knowing their experience about online voting system. We have attached the questionnaires and feedback from users in the **Appendix** section. Performance evaluation of this voting app from user-end have also been attached in **Appendix** section. We have also attached a graph of positive and negative responses about the voting system.

## 6 Conclusion

With a few recommendations for best practices in the future, this section assesses and concludes the research study presented in this section. However, there are still certain obstacles that can be removed in the upcoming applications of this work and the execution of improved suggestions.

### 6.1 Summary of voting mechanism

This article discusses the benefits and challenges of developing an online voting app. The verification process includes face recognition using MobileFaceNet and a haar-cascade classifier, stored in the database. The device fingerprint is used for voting purposes, as biometric data cannot be shared outside the mobile device. The app includes time selection, vote counting, and blocking duplicate votes. The voter registration process includes OTP validation and a mobile number filter to prevent duplicate registrations.

### 6.2 Scope and limitation

This online voting management system can be applied to various types of elections, such as municipal councilor selection or class representative selection. However, the system has limitations. Because implementation of an online voting system is highly needed but enough knowledge about this technique is missing from the user. Spreading that kind of knowledge requires more time before implementation. Despite cybersecurity measures, new threats can emerge. Continuous vigilance and adaptation of security measures are essential to counter potential attacks. We have contributed hash algorithm for specific data integrity purposes. But the hash algorithm has been broken for decades. One viable alternative is to employ a more secure hashing algorithm, such as SHA-3 (Keccak), which was selected as the winner of the NIST hash function competition in 2012 and is considered highly secure. Additionally, one could explore the use of cryptographic hash functions like BLAKE2 or SHA-512, which offer higher levels of security compared to SHA-256.

### 6.3 Future research direction

Future developments of the online voting management system include text recognition of voter ID number and date of birth from a photograph of the voter identity card. Additionally, implementing a low-cost biometric fingerprint scanner will be a significant achievement for the system's security. Alternative authentication options for users without biometric-capable devices could further enhance inclusivity. Our contribution is to use RSA encryption and decryption technology for data integrity and security. But nowadays, for better data integrity and security purposes, one can try to build the system with Homomorphic encryption because it allows computation on encrypted data without decrypting it.

RETRACTED

## Funding

There was no explicit support for this study from the government, industry, or non-profit funding organization. It was self-funded research.

## Additional information

No additional information is available for this paper.

## Data availability statement

Data associated with this study has not been deposited into a publicly available repository because voter's information has been used as the data for training and testing of various verification techniques which should be kept confidential.

## CRediT authorship contribution statement

**Kazi Naimur Rahman:** Writing – review & editing, Writing – original draft, Visualization, Validation, Software, Resources, Project administration, Methodology, Investigation, Funding acquisition, Formal analysis, Data curation, Conceptualization. **Monowar Wadud Hridoy:** Supervision. **Md Mizanur Rahman:** Supervision. **Md Rifatul Islam:** Validation, Formal analysis, Data curation, Visualization, Writing – original draft. **Semonti Banik:** Visualization, Validation, Formal analysis, Data curation, Writing – original draft.

## Declaration of competing interest

The authors declare that they have no known competing financial interests or personal relationships that could have appeared to influence the work reported in this paper.

## APPENDIX

Video of Online Voting System:

https://drive.google.com/file/d/1YeqsNhPr9EVa3kLvKYvVo4gvS0GNLd9R/view?usp=sharing

Graphical User Interface (GUI) of Online Voting System:

https://docs.google.com/document/d/1eAPHNXiSatuiuY69cPDGkvH6Lv4Kt6c0dMLS_41Vn9I/edit?usp=sharing

### Performance Evaluation Questionnaire

https://docs.google.com/spreadsheets/d/18daZoTNcDYHpnsheNDNBhIf1Ly_kk9V5SONEFQcrDyU/edit?usp=sharing
